# Effect of Different General Anesthesia Methods on the Prognosis of Patients with Breast Cancer after Resection: A Systematic Review and Meta-analysis

**DOI:** 10.1155/2022/6846079

**Published:** 2022-06-28

**Authors:** Rui Lv, Chunli Zhang, Yuyuan Huang, Peng Xiao

**Affiliations:** ^1^Department of Anesthesiology, Sanya Women and Children's Hospital Managed by Shanghai Children's Medical Center, Sanya, 572000 Hainan, China; ^2^Department of Anesthesiology, The Second Affiliated Hospital of Hainan Medical University, Haikou, 570311 Hainan, China; ^3^Department of Anesthesiology, Hainan Provincial Hospital of Chinese Medicine, Haikou, 570203 Hainan, China

## Abstract

**Background:**

The effect of total intravenous anesthesia (TIVA) and inhalation anesthesia (IA) on the prognosis of breast cancer patients has been controversial. The study is aimed at exploring the effects of different anesthesia methods on the postoperative prognosis of breast cancer patients.

**Methods:**

Literature retrieval was conducted in PubMed, EMBASE, MEDLINE, Embase, CENTRAL, and CNKI databases. The literature topic was to compare the effects of TIVA and IA on the prognosis of patients undergoing breast cancer resection. Two researchers extracted data from the literature independently. This study included randomized controlled trials that evaluated for risk of bias according to the “Risk assessment Tool for Bias in Randomized Trials” in the Cochrane Manual. The Newcastle-Ottawa Scale (NOS) was used to assess the risk of bias in observational studies. The chi-square test was used for the heterogeneity test. Publication bias was assessed using funnel plots and Egger's test. If heterogeneity existed between literature, subgroup analysis and sensitivity analysis were used to explore the source of heterogeneity. Sensitivity analysis was performed by excluding low-quality and different-effect models. Data were statistically analyzed using the Cochrane software RevMan 5.3. Hazard ratio (HR) and 95% confidence interval (CI) were used for statistical description.

**Results:**

Seven literatures were selected for meta-analysis. There were 9781 patients, 3736 (38.20%) receiving TIVA and 6045 (61.80%) receiving inhalation anesthesia. There was no significant difference in overall survival (OS) between TIVA and IA breast cancer patients (HR = 1.05, 95% CI (0.91, 1.22), *Z* = 0.70, *P* = 0.49). There was no difference in the literature (*χ*^2^ = 6.82, *P* = 0.34, *I*^2^ = 12%), and there was no obvious publication bias. There was no significant difference in recurrence-free survival (RFS) between TIVA and IA patients (HR = 0.95, 95% CI (0.79, 1.13), *Z* = 0.61, *P* = 0.54). There was no heterogeneity in the literature (*χ*^2^ = 5.23, *P* = 0.52, *I*^2^ = 0%), and there was no significant publication bias.

**Conclusion:**

There is no significant difference in OS and RFS between TIVA and IA patients during breast cancer resection. The prognostic effects of TIVA and IA were similar.

## 1. Introduction

Breast cancer is one of the most common malignant tumours and the leading cause of female cancer death. Surgical resection is the main treatment plan [1], but the stress, anesthesia, and narcotic drugs caused by surgery adversely affect postoperative recovery and anticancer immunity [2]. General anesthesia is the primary anesthesia method for breast surgery, including total intravenous anesthesia (TIVA) and inhalation anesthesia (IA) [3]. These two general anesthesia methods have different side effects on patients and immune status because of the differences in drug administration and drug use [4]. The choice of general anesthesia may affect the postoperative rehabilitation and prognosis of patients.

A previous meta-analysis [5] illustrated that TIVA could reduce the recurrence rate of malignant tumours and prolong the OS and RFS of patients. Both in vivo and in vitro studies have confirmed that volatile anesthetic drugs promote the proliferation, invasion, and migration of malignant tumour cells [6–9]. At the same time, propofol used in TIVA can inhibit the proliferation and metastasis of malignant tumour cells [10]. In breast cancer, the influence of TIVA and IA on the prognosis of breast cancer patients has been controversial. Previous research results fail to show a consistent trend. Some studies [11] indicated that intravenous anesthesia could improve the immune function of patients with breast cancer. The postoperative recurrence-free survival rate of patients with inhalation anesthesia was worse than that of patients with intravenous anesthesia. However, some studies [12] have shown no difference between the two anesthesia methods in the overall survival or relapse-free survival of breast cancer.

Based on the above controversy, this study is aimed at exploring the impact of TIVA and IA on the prognosis of breast cancer patients after resection through meta-analysis.

## 2. Materials and Methods

### 2.1. Bibliography Retrieval

The keywords included intravenous anesthesia, propofol, propofol-based intravenous anesthesia, inhalation anesthesia, breast cancer, breast surgery, mastectomy, and radical mastectomy. The literature was searched in PubMed, EMBASE, MEDLINE, Embase, CENTRAL database, and CNKI database according to the search terms. The documents were written in English and Chinese. The date of the literature search was March 5, 2022.

### 2.2. Literature Screening

Inclusion criteria are as follows: (1) The subjects were female patients with breast cancer; (2) the control group was set up in the study; (3) TIVA was implemented in the experimental group, and IA was implemented in the control group; (4) the observed indexes of the study included at least one of the recurrence-free survival (RFS) or overall survival of patients with breast cancer after operation; (5) research types included a randomized controlled trial (RCT) and observational study; and (6) the statistical data in the literature could calculate the value of hazard ratio (HR) and 95% confidence interval (CI).

Literature exclusion criteria are as follows: (1) other anesthesia methods were used to assist surgical treatment; (2) the subjects selected in the literature were complicated with other tumours; (3) no control group was set; (4) the baseline data of the control group and the experimental group were poorly balanced; (5) the literature data was incomplete and could not be supplemented by contacting the literature author.

### 2.3. Document Data Sorting

Lv and Xiao independently extracted the data and information from the literature. Two researchers used plot-digitizer software to extract graphic data information. The authors were contacted by email to request relevant data not shown in the literature. Two researchers cross-examined each other's data. If there were differences between the two authors, negotiation could reach an agreement.

### 2.4. Literature Quality Evaluation

Lv and Zhang evaluated the literature quality. According to the “bias risk assessment tool of randomized trials” in the Cochrane Manual, the bias risk assessment of RCTs was carried out. The evaluation contents included five aspects: the bias in the process of randomization, the bias from the established intervention measures, the bias from the lack of outcome data, the bias of outcome measurement, and the bias of selective reporting results. The literature was divided into “low risk of bias,”, “some risks,” and “high risk of bias.” In the current study, the Newcastle-Ottawa Scale (NOS) was used to assess the risk of bias in observational studies. The contents included the selection of subjects (4 points), comparability between groups (2 points), and exposure factor measurement (3 points), a total of 9 points. In case of inconsistency in the judgment results of literature quality, two researchers reached an agreement after discussion. The two researchers compared the evaluation results after completing the literature quality evaluation. If there were differences, the two authors reached an agreement through discussion.

### 2.5. Heterogeneity Test and Publication Bias Test

The chi-square test was used for the heterogeneity test. When *I*^2^ > 50% or *P* < 0.1, it was considered that there was heterogeneity among published literatures, and a random effect model was used. When *I*^2^ ≤ 50% or *P* ≥ 0.1, there was no heterogeneity among published literatures, and the fixed-effect model was adopted. Funnel plots and Egger's test were used for the publication bias test.

### 2.6. Subgroup Analysis and Sensitivity Analysis

If there was heterogeneity between literature, subgroup analysis and sensitivity analysis were used to explore the source of heterogeneity. Sensitivity analysis was carried out by excluding low-quality and different effect models.

### 2.7. Statistical Method

This study used the Cochrane software RevMan 5.3 statistical analysis of the data. HR value and 95% CI were used for statistical description. Two-way *P* < 0.05 indicates statistically significant.

## 3. Results

### 3.1. Retrieval Results and Literature Quality Evaluation

According to the relevant subject words, this study retrieved 1846 articles about the impact of TIVA and IA on the prognosis of breast cancer patients after resection. According to the literature screening criteria, 7 literatures were further selected for meta-analysis. The flow chart of literature screening is shown in Figure 1. A total of 9781 breast cancer resection patients were included in the 7 articles, including 3736 (38.20%) patients receiving TIVA and 6045 (61.80%) patients receiving inhalation anesthesia. The risk assessment of literature bias is shown in Table 1.

### 3.2. Effects of TIVA and IA on Postoperative OS in Patients with Breast Cancer

Seven articles compared OS in patients with TIVA and IA breast cancer after the operation. There was no heterogeneity between the literatures (*χ*^2^ = 6.82, *P* = 0.34, *I*^2^ = 12%). The fixed-effect model was used to merge the effects (HR = 1.05; 95% CI (0.91, 1.22), test of overall effect *Z* = 0.70 (*P* = 0.49), see Figure 2). The analysis showed no significant difference in OS between TIVA and IA breast cancer patients. The funnel plot and Egger's test were showed that the scatter points were roughly symmetrical within the confidence interval, and there was no obvious publication bias (*P* > 0.05), as shown in Figure 3.

### 3.3. Effects of TIVA and IA on Postoperative RFS in Patients with Breast Cancer

Seven articles compared RFS in patients with TIVA and IA breast cancer. There was no heterogeneity between the literatures (*χ*^2^ = 5.23, *P* = 0.52, *I*^2^ = 0%). The fixed-effect model was used to merge the effects (HR = 0.95; 95% CI (0.79, 1.13), test of overall effect *Z* = 0.61 (*P* = 0.54), see Figure 4). The analysis showed no significant difference in RFS between TIVA and IA breast cancer patients. The funnel plot and Egger's test were indicated that the scatter points were roughly symmetrical within the confidence interval, and there was no obvious publication bias (*P* > 0.05), as shown in Figure 5.

## 4. Discussion

This meta-analysis recruited seven randomized controlled trials to compare the effects of TIVA and IA on the prognosis of patients with breast cancer after resection. We found no statistically significant difference in OS and RFS between TIVA and IA breast cancer patients. The results from previous studies are consistent with our analysis. Cho et al. [11] suggested that the analgesic effects of TIVA and IA were similar. TIVA could increase the proportion of NK cells in the blood of breast cancer patients after the operation and promote the immune function of breast cancer patients, thus reducing the recurrence rate of breast cancer. Hong et al. [13] showed that TIVA and IA had similar effects on OS in patients with malignant tumours through retrospective analysis. These tumours included breast cancer, liver cancer, lung cancer, gastric cancer, and colon cancer. Through retrospective analysis, Huang et al. [12] compared the prognosis of 632 breast cancer patients receiving IA and 334 breast cancer patients receiving TIVA. They pointed out no statistically significant difference in the 5-year survival and recurrence rate of breast cancer patients receiving the two anesthesia methods. Kim et al. [14] considered that TIVA and IA have similar effects on the prognosis of breast cancer patients. Yan et al. [15] showed that IA could increase VEGF expression in the serum of breast cancer patients, but there was no significant difference in the recurrence rate and survival rate of breast cancer. Yan et al. [16] showed no significant difference between TIVA and IA in myeloid-derived suppressor cells (MDSCs), overall survival rate, and recurrence rate after resection of breast cancer patients. Yoo et al. [2] considered that TIVA or IA had no significant effect on RFS and OS in patients undergoing breast cancer resection.

A meta-analysis pointed out that TIVA could reduce the recurrence of malignant tumours and prolong OS and RFS [5]. Meanwhile, various cancer types, such as breast cancer, non-small-cell lung cancer, colon cancer, rectal cancer, and gastric cancer, were included in that study. Furthermore, researchers observed a magnified effect in malignant surgery. With prolonged operation time, TIVA might increase the prognosis of patients. Yap et al. [5] also pointed out that TIVA could improve RFS in patients with breast cancer but had no effect on OS compared with IA. The possible reason for this phenomenon is that propofol used in TIVA can inhibit tumour metastasis. At the same time, volatile gas anesthetics may promote tumour cell metastasis and proliferation and inhibit cancer cell apoptosis [6–10].

A previous meta-analysis [17] has shown that the analgesic effect of intravenous anesthesia is inferior to inhalation anesthesia and can reduce the incidence of postoperative vomiting. Intravenous anesthesia is superior to inhalation anesthesia in maintaining anticancer immune status. Its potential mechanism is that propofol reduces IL-6 while retaining NKCC and NLR in the blood. In this current study, we speculate that propofol may potentially benefit the long-term prognosis of breast cancer after surgery. However, we did not find any difference in the prognosis of patients under intravenous anesthesia and inhalation anesthesia.

Studies have shown that propofol is associated with a higher relapse-free survival rate after breast surgery in malignant tumours with or without breast cancer. Still, it cannot reduce recurrence or prolong overall survival [18]. It is also pointed out that propofol-based intravenous anesthesia has advantages over inhalation anesthesia in reducing long-term recurrence and metastasis of tumours [19]. More multicenter, large sample size prospective randomized controlled trials are needed to explore the potential protective effect of propofol intravenous anesthesia on the long-term prognosis of breast cancer patients.

In conclusion, in breast cancer resection, there was no significant difference in OS and RFS between breast cancer resection patients who received TIVA versus IA. TIVA and IA have similar prognostic effects on patients.

## Figures and Tables

**Figure 1:** Flow chart of literature screening.

**Figure 2:** Forest map: comparison of postoperative OS between TIVA and IA breast cancer patients. TIVA: total intravenous anesthesia; IA: inhalation anesthesia; OS: overall survival.

**Figure 3:** Funnel diagram: comparison of postoperative OS between TIVA and IA breast cancer patients. TIVA: total intravenous anesthesia; IA: inhalation anesthesia; OS: overall survival.

**Figure 4:** Forest map: comparison of postoperative OS between TIVA and IA breast cancer patients. TIVA: total intravenous anesthesia; IA: inhalation anesthesia; RFS: recurrence-free survival.

**Figure 5:** Funnel diagram: comparison of postoperative OS between TIVA and IA breast cancer patients. TIVA: total intravenous anesthesia; IA: inhalation anesthesia; RFS: recurrence-free survival.

**Table 1:** Risk of bias assessment.

Study	Study design	No. of patients		Risk of bias assessment
		TIVA	IA	
Cho et al. [11]	RCT	25	25	Low risk of bias
Hong et al. [13]	Retrospective	154	475	NOS score 7
Huang et al. [12]	Retrospective	334	632	NOS score 6
Kim et al. [14]	Retrospective	56	2589	NOS score 7
Yan et al. [15]	RCT	40	40	Low risk of bias
Yan et al. [16]	RCT	42	38	Low risk of bias
Yoo et al. [2]	Retrospective	3085	2246	NOS score 7

Note: TIVA: total intravenous anesthesia; IA: inhalation anesthesia; NOS: Newcastle-Ottawa Scale.

## Data Availability

The data used to support the findings of this study are included within the article.
